# Novel Type I Half Logistic Burr-Weibull Distribution: Application to COVID-19 Data

**DOI:** 10.1155/2022/1444859

**Published:** 2022-08-18

**Authors:** Huda M. Alshanbari, Omalsad Hamood Odhah, Ehab M. Almetwally, Eslam Hussam, Mutua Kilai, Abdal-Aziz H. El-Bagoury

**Affiliations:** ^1^Department of Mathematical Sciences, College of Science, Princess Nourah bint Abdulrahman University, P.O. Box 84428, Riyadh 11671, Saudi Arabia; ^2^Department of Statistics, Faculty of Business Administration, Delta University of Science and Technology, Egypt; ^3^The Scientific Association for Studies and Applied Research, Al Manzalah 35646, Egypt; ^4^Department of Mathematics, Helwan University, Faculty of Science, Cairo, Egypt; ^5^Department of Mathematics, Pan African Institute of Basic Science Technology and Innovation, Nairobi, Kenya; ^6^Basic Science Department, Higher Institute of Engineering and Technology, El-Mahalla El-Kubra, Egypt

## Abstract

In this work, we presented the type I half logistic Burr-Weibull distribution, which is a unique continuous distribution. It offers several superior benefits in fitting various sorts of data. Estimates of the model parameters based on classical and nonclassical approaches are offered. Also, the Bayesian estimates of the model parameters were examined. The Bayesian estimate method employs the Monte Carlo Markov chain approach for the posterior function since the posterior function came from an uncertain distribution. The use of Monte Carlo simulation is to assess the parameters. We established the superiority of the proposed distribution by utilising real COVID-19 data from varied countries such as Saudi Arabia and Italy to highlight the relevance and flexibility of the provided technique. We proved our superiority using both real data.

## 1. Introduction

One of the fundamental objectives of statistics is to develop appropriate statistical models for natural and real-world events defined by well-established statistical probability distributions. This is one of the primary functions of statistics.

In this instance, probability distributions are used to characterise the unpredictability and potential hazard of the life event under investigation. As a result of the extreme difficulty of reproducing real-life events using ordinary probability distributions, several probability distributions have been developed.

Using probability distributions is one of the most important aspects of statistic to model real-world events. Knowable probability distributions are used to model uncertain and risky natural phenomena.

Due to the complexity and variety of natural phenomena, several probability distributions are derived. Nonetheless, identified probability distributions are incapable of accurately representing data for certain natural phenomena. These are useful for extending and altering generalized probability distributions.

Due to the widespread availability of additional parameters, generalized probability distributions have advanced. By adding a few parameters to well-known probability distributions, their suitability for data from natural phenomena was improved, as was the precision of the distribution tail shape description.

Oftentimes, the known and accessible probability distributions are inadequate to accurately represent and characterise information resulting from certain natural phenomena. As a result of the modifications and expansions that have taken place, the generalized probability distributions are changed and enlarged.

The world has been ravaged by a variety of pandemics and diseases throughout the whole of human existence. Other recent coronavirus outbreaks include COVID-19, which arose last year and has been classified a global epidemic. This outbreak is historically regarded as one of the most terrifying infectious illnesses in human history.

COVID-19's worldwide growth has been inhibited as a result of the deployment of “strict” safety procedures by the vast majority of nations.

Various additional measures, such as total restrictions on commerce and shorter business and nighttime school hours, have also been implemented. Among other features, a complete mathematical and statistical model was constructed and evaluated to predict the course of future COVID-19-related disorders.

Researchers have taken an interest in presenting new wide families of continuous univariate distributions and their successful application during the course of the last two decades. By adding one or more additional shape components to a baseline distribution, a growing interest has been sparked in the production of new classes of distributions. These characteristics make the produced distribution more adaptable and accurate for evaluating tail behaviour.

However, there are still a great number of significant instances in which real-world data does not conform to any classical or conventional probability model. In latest days, several sorts of families have been introduced.

Among the most notable generators are the following: an innovative method for integrating a parameter into a family of distributions, which consists of merging the distributions themselves (see [1], beta-*G* by [2], logistic-*X* by [3–10], the transmuted odd Fréchet-*G* family by [11], and Burr X Exponential-*G* family by [12], among others.

Both the probability density function (PDF) and the cumulative distribution function (CDF) of the Weibull distribution, together with the parameter *β*, *δ* > 0, are the following:

(1) $$\begin{array}{c} G\left(x;\beta ,\delta \right)=1-e^{-\delta x^{\beta }},\;x\geq 0,\beta ,\delta >0, \end{array}$$

(2) $$\begin{array}{c} g\left(x;\delta \right)=\beta \delta x^{\beta -1}e^{-\delta x^{\beta }},\;x,\delta >0. \end{array}$$

[13] presented a novel generator based on the Burr *X* random variable, which is well-known *X* − *G* family of distributions. [14] made a novel family of continuous distributions with an extra positive parameter *λ* > 0 called the type I half logistic-*G* (TIHL − *G*) family. Recently, a new generator based on theTIHL − *G*family and Burr*X* − *G*family constructed a new family called the type I half logistic Burr*X* − *G*(TIHLBX − *G*)family of distributions by Algarni et al. [15]. This series is more versatile and attracts a larger range of health modeling field purposes. The CDF and PDF of TIHLBX − *G* family of distributions, respectively, are given by

(3) $$\begin{array}{c} F\left(x;\lambda ,\alpha ,\delta \right)=\frac{1-{\left\{1-{\left[1-e^{-{\left(G\left(x;\delta \right)/\bar{G}\left(x;\delta \right)\right)}^{2}}\right]}^{\alpha }\right\}}^{\lambda }}{1+{\left\{1-{\left[1-e^{-{\left(G\left(x;\delta \right)/\bar{G}\left(x;\delta \right)\right)}^{2}}\right]}^{\alpha }\right\}}^{\lambda }},\\ f\left(x;\lambda ,\alpha ,\delta \right)=\frac{4\lambda \alpha g\left(x;\delta \right)}{\bar{G}{\left(x;\delta \right)}^{3}}G\left(x;\delta \right)e^{-{\left(G\left(x;\delta \right)/\bar{G}\left(x;\delta \right)\right)}^{2}}{\left[1-e^{-{\left(G\left(x;\delta \right)/\bar{G}\left(x;\delta \right)\right)}^{2}}\right]}^{\alpha -1},\\ {\left\{1-{\left[1-e^{-{\left(G\left(x;\delta \right)/\bar{G}\left(x;\delta \right)\right)}^{2}}\right]}^{\alpha }\right\}}^{\lambda -1}{\left\{1+{\left\{1-{\left[1-e^{-{\left(G\left(x;\delta \right)/\bar{G}\left(x;\delta \right)\right)}^{2}}\right]}^{\alpha }\right\}}^{\lambda }\right\}}^{-2}, \end{array}$$

where *g*(*x*; *δ*) and *G*(*x*; *δ*) are the baseline distribution's PDF and CDF in the given parameter vector *δ*.

As a consequence of this, the composite distribution that emerges as a consequence of this procedure will only include a total of four parameters. These four parameters will be comprised of two parameters derived from the baseline distribution, which is the Weibull distribution, and two parameters derived from the TIHLB-*G* family of distributions.

The exponential distribution is one of the most important probability models in the science of statistics as well as in other fields of inquiry; it is comprised of distributions such as the Rayleigh distribution and the exponential distribution. One of the most essential components of the Weibull distribution, the exponential distribution, is regarded as one of the most influential types of probability models.

A number of efforts have been made in the past to broaden the scope of this distribution, for example, see [16–18] and [19], which are some of the most well-known pieces of literary composition.

However, when a more versatile family of distributions is utilised, the modelling capability of the flexible Weibull distribution may be boosted; it is one of the challenges that our current study tackles. More articles have been addressed, including the new Weibull distribution expansion (see [20–25], etc.).

The purpose of this study is to build a four-parameter TIHLB Weibull distribution, establish its different attributes, estimate its unknown parameters, and illustrate its strength via the use of COVID-19 data in a practical applications. When it comes to PDF, the TIHLBW distribution is quite adaptable; it may be positive skewed, negative slanted, and symmetrical, and it can allow for more versatility in the tails. The TIHLBW distribution features a PDF that is quite versatile; it may be positively skewed, negatively skewed, or symmetric, and it can allow for more flexibility in the tails of the distribution.

It is capable of simulating hazard rates that are monotonically declining, growing, bathtub, upside down bathtub, and reversed-J in nature, among other things. Moreover, the distribution has a closed-form CDF and is relatively simple to handle, which makes it a good choice for usage in a variety of domains such as life testing, durability, biological investigations, and survival analysis.

Using actual data, three instances demonstrate that the suggested distribution is quite comparable with certain existing distributed models.

An innovative form of the Weibull distribution is referred to as the TIHLBX Weibull distribution. This distribution may also be referred to as the TIHLBW distribution. We have built a novel distribution in the hopes of boosting its versatility and garnering a wider variety of uses in dependability, economics, biopsychosocial issues related, and other study domains.

The following is the structure of the rest of this paper. In Section 2, we find out how to calculate the TIHLBW distribution. TIHLBW distribution has a number of mathematical features, which we will analyse in Section 3. In Section 4, we derive an estimate technique MKITL distribution using the MKITL estimation technique. In Section 5, we derive the results of a simulations of the TIHLBW probability distribution. Using actual data analysis, we were able to acquire three applications in Section 6.  Section 7 provides a summary and conclusion to the work.

## 2. TIHLBW Distribution

In the field of statistics, one of the most significant challenges is deciding which probability distribution is the best suitable to use when trying to draw conclusions from certain sets of data. Because of this factor, academics in the recent past have put in a significant amount of work to build distributions. There is a wide range of univariate continuous distributions and their applications in modelling real-world data that may be found in the body of academic research.

Many other classes of distributions have been produced in recent years. These distributions have been created by adding an additional shape parameter or parameters to an existing distribution in order to make the distribution more flexible. Studying the actions of tails becomes more interesting as a result.

Weibull, Rayleigh, and exponential distributions are some of the most commonly used distributions for modeling lifetime data by researchers.

When the exponential distribution is taken into account, it only demonstrates constant danger shapes; when the Rayleigh distribution is taken into consideration, it only demonstrates a rising hazard function shape. When modelling data that may be categorised as either constant, decreasing, or rising hazard shape, the Weibull distribution has been the distribution that has been used the most often. The Weibull distribution has a flaw in that it is not ideal for handling data that are characterised by nonmonotonic hazard shapes.

This is one of the distribution's shortcomings. The vast majority of lifetime data exhibits the characteristic of having nonmonotonic hazard forms.

Analyse the Weibull distribution using the CDF and PDF values that have been provided (for *x* > 0) by Equations (1) and (2), respectively. By entering the CDF of the Weibull distribution into the TIHLBW distribution, we can define the CDF of the TIHLBW distribution (4), to provide an example:

(4) $$\begin{array}{c} F\left(x;\Omega \right)=\frac{1-{\left\{1-{\left[1-e^{-{\left(e^{\delta x^{\beta }}-1\right)}^{2}}\right]}^{\alpha }\right\}}^{\lambda }}{1+{\left\{1-{\left[1-e^{-{\left(e^{\delta x^{\beta }}-1\right)}^{2}}\right]}^{\alpha }\right\}}^{\lambda }}, \end{array}$$

(5) $$\begin{array}{c} f\left(x;\Omega \right)=4\lambda \alpha \beta \delta x^{\beta -1}e^{2\delta x^{\beta }}\left(1-e^{-\delta x^{\beta }}\right)e^{-{\left(e^{\delta x^{\beta }}-1\right)}^{2}}{\left[1-e^{-{\left(e^{\delta x^{\beta }}-1\right)}^{2}}\right]}^{\alpha -1}{\left\{1-{\left[1-e^{-{\left(e^{\delta x^{\beta }}-1\right)}^{2}}\right]}^{\alpha }\right\}}^{\lambda -1}{\left\{1+{\left\{1-{\left[1-e^{-{\left(e^{\delta x^{\beta }}-1\right)}^{2}}\right]}^{\alpha }\right\}}^{\lambda }\right\}}^{-2}, \end{array}$$

where *Ω* is vector of parameters (*α*, *λ*, *δ*, *λ*). For more shape density of this model, see Figure 1.

The hazard rate (HR) function of the TIHLBW distribution is shown as

(6) $$\begin{array}{c} \tau \left(x;\Omega \right)=\frac{2\lambda \alpha \beta \delta x^{\beta -1}e^{2\delta x^{\beta }}\left(1-e^{-\delta x^{\beta }}\right)e^{-{\left(e^{\delta x^{\beta }}-1\right)}^{2}}{\left[1-e^{-{\left(e^{\delta x^{\beta }}-1\right)}^{2}}\right]}^{\alpha -1}}{\left[1-{\left[1-e^{-{\left(e^{\delta x^{\beta }}-1\right)}^{2}}\right]}^{\alpha }\right]\left\{1+{\left[1-{\left[1-e^{-{\left(e^{\delta x^{\beta }}-1\right)}^{2}}\right]}^{\alpha }\right]}^{\lambda }\right\}}. \end{array}$$

For more shape HR of this model, see Figure 2.

### 2.1. Useful Expansion

*f*, (*x*) and *F*, (*x*) expansions are made easier with the following findings (*x*). If |*z*| < 1 is a real noninteger and *b* > 0 is a real noninteger, then the power series shown below holds. The subsequent outcomes are beneficial for extensions of *f*(*x*) and *F*(*x*).

(7) $$\begin{array}{c} f\left(x;\lambda ,\alpha ,\delta \right)=4\lambda \alpha \overset{\infty }{\underset{i,j,k=0}{\sum }}{\left(-1\right)}^{j+k}\left(\begin{array}{c} -2\\ i \end{array}\right)\frac{\gamma \left(\lambda \left(i+1\right)\right)\gamma \left(\alpha \left(j+1\right)\right)}{j!k!\gamma \left(\lambda \left(i+1\right)-j\right)\gamma \left(\alpha \left(j+1\right)-k\right)}\times \overset{\infty }{\underset{m=0}{\sum }}\frac{{\left(-1\right)}^{m}{\left(k+1\right)}^{m}}{m!}\frac{g\left(x;\delta \right)}{\bar{G}{\left(x;\delta \right)}^{2m+3}}G{\left(x;\delta \right)}^{2m+1}. \end{array}$$

Using the generalized binomial expansion, we can rewrite the PDF as follows:

(8) $$\begin{array}{c} f_{\text{TIHLBW}}\left(x;\lambda ,\alpha ,\delta \right)=\overset{\infty }{\underset{m,d=0}{\sum }}\varpi_{m,d}\pi_{\left(2\left(m+1\right)+d\right)}\left(x\right), \end{array}$$

where

(9) $$\begin{array}{c} \varpi_{m,d}=\overset{\infty }{\underset{i,j,k=0}{\sum }}{\left(-1\right)}^{j+k+m}\left(\begin{array}{c} -2\\ i \end{array}\right)\frac{4\lambda \alpha \gamma \left(\lambda \left(i+1\right)\right)\gamma \left(\alpha \left(j+1\right)\right)}{j!k!m!d!\gamma \left(\lambda \left(i+1\right)-j\right)\gamma \left(\alpha \left(j+1\right)-k\right)}\times \frac{{\left(k+1\right)}^{m}\gamma \left(2m+d+3\right)}{\gamma \left(2m+3\right)\left(2\left(m+1\right)+d\right)}, \end{array}$$

and *π*_(2(*m* + 1) + *d*)_(*x*) = (2(*m* + 1) + *d*)*βδx*^*β*−1^*e*^−*δx*^*β*^^(1 − *e*^−*δx*^*β*^^)^2*m*+*d*+1^ is the expo-*G* PDF with power parameter (2(*m* + 1) + *d*). Thus, several mathematical and statistical properties of the TIHLBW distribution can be determined obviously from those of exp-Weibull distribution.

## 3. Maximum Likelihood Estimation

In addition to having beneficial qualities, the MLEs may be employed in the construction of confidence intervals and regions, as well as in test statistics. In this study, we use solely complete samples to derive the maximum likelihood estimates (MLEs) of the parameters of the TIHLBW distribution. Let *x*_1_, ⋯, *x*_*n*_ be a random sample of size *n* from the TIHLBW distribution given by (5). Let *Ω* = (*α*, *λ*, *δ*, *λ*)^*T*^ be vector of parameters. The likelihood function is given by

(10) $$\begin{array}{c} Ł\left(\Omega \right)=4^{n}\lambda^{n}\alpha^{n}\beta^{n}\delta^{n}e^{2\delta \overset{n}{\underset{i=1}{\sum }}x_{i}^{\beta }}e^{-\overset{n}{\underset{i=1}{\sum }}{\left(e^{\delta x_{i}^{\beta }}-1\right)}^{2}}\overset{n}{\underset{i=1}{\prod }}x_{i}^{\beta -1}\left(1-e^{-\delta x_{i}^{\beta }}\right){\left[1-e^{-{\left(e^{\delta x_{i}^{\beta }}-1\right)}^{2}}\right]}^{\alpha -1}\times \overset{n}{\underset{i=1}{\prod }}{\left\{1-{\left[1-e^{-{\left(e^{\delta x_{i}^{\beta }}-1\right)}^{2}}\right]}^{\alpha }\right\}}^{\lambda -1}{\left\{1+{\left\{1-{\left[1-e^{-{\left(e^{\delta x_{i}^{\beta }}-1\right)}^{2}}\right]}^{\alpha }\right\}}^{\lambda }\right\}}^{-2}. \end{array}$$

The log-likelihood function is given by

(11) $$\begin{array}{c} \ell \left(\Omega \right)=n\left[\ln\left(4\right)+\ln\left(\lambda \right)+\ln\left(\alpha \right)+\ln\left(\beta \right)+\ln\left(\delta \right)\right]+\left(\beta -1\right)\overset{n}{\underset{i=1}{\sum }}\ln\left(x_{i}\right)-\overset{n}{\underset{i=1}{\sum }}{\left(e^{\delta x_{i}^{\beta }}-1\right)}^{2}+\overset{n}{\underset{i=1}{\sum }}\ln\left(1-e^{-\delta x^{\beta }}\right)+2\delta \overset{n}{\underset{i=1}{\sum }}x_{i}^{\beta }-2\overset{n}{\underset{i=1}{\sum }}\ln\left\{1+{\left\{1-{\left[1-e^{-{\left(e^{\delta x_{i}^{\beta }}-1\right)}^{2}}\right]}^{\alpha }\right\}}^{\lambda }\right\}+\left(\lambda -1\right)\overset{n}{\underset{i=1}{\sum }}\ln\left\{1-{\left[1-e^{-{\left(e^{\delta x_{i}^{\beta }}-1\right)}^{2}}\right]}^{\alpha }\right\}+\left(\alpha -1\right)\overset{n}{\underset{i=1}{\sum }}\ln\left[1-e^{-{\left(e^{\delta x_{i}^{\beta }}-1\right)}^{2}}\right]. \end{array}$$

After obtaining the initial partial derivatives of (11) with regard to *α*, *λ*, *δ*, *λ* and then equating each partial derivative to 0, we are able to arrive at the desired result.

(12) $$\begin{array}{c} \frac{\partial \ell \left(\Omega \right)}{\partial \lambda }=\frac{n}{\lambda }+\overset{n}{\underset{i=1}{\sum }}\ln\left\{1-{\left[1-e^{-{\left(e^{\delta x_{i}^{\beta }}-1\right)}^{2}}\right]}^{\alpha }\right\}-2\overset{n}{\underset{i=1}{\sum }}\frac{{\left\{1-{\left[1-e^{-{\left(e^{\delta x_{i}^{\beta }}-1\right)}^{2}}\right]}^{\alpha }\right\}}^{\lambda }\ln\left\{1-{\left[1-e^{-{\left(e^{\delta x_{i}^{\beta }}-1\right)}^{2}}\right]}^{\alpha }\right\}}{1+{\left\{1-{\left[1-e^{-{\left(e^{\delta x_{i}^{\beta }}-1\right)}^{2}}\right]}^{\alpha }\right\}}^{\lambda }},\\ \frac{\partial \ell \left(\Omega \right)}{\partial \alpha }=\frac{n}{\alpha }+2\lambda \overset{n}{\underset{i=1}{\sum }}\frac{{\left[1-e^{-{\left(e^{\delta x_{i}^{\beta }}-1\right)}^{2}}\right]}^{\alpha }\ln\left[1-e^{-{\left(e^{\delta x_{i}^{\beta }}-1\right)}^{2}}\right]{\left\{1-{\left[1-e^{-{\left(e^{\delta x_{i}^{\beta }}-1\right)}^{2}}\right]}^{\alpha }\right\}}^{\lambda -1}}{1+{\left\{1-{\left[1-e^{-{\left(e^{\delta x_{i}^{\beta }}-1\right)}^{2}}\right]}^{\alpha }\right\}}^{\lambda }}-\left(\lambda -1\right)\overset{n}{\underset{i=1}{\sum }}\frac{\ln\left[1-e^{-{\left(e^{\delta x_{i}^{\beta }}-1\right)}^{2}}\right]{\left[1-e^{-{\left(e^{\delta x_{i}^{\beta }}-1\right)}^{2}}\right]}^{\alpha }}{1-{\left[1-e^{-{\left(e^{\delta x_{i}^{\beta }}-1\right)}^{2}}\right]}^{\alpha }}+\overset{n}{\underset{i=1}{\sum }}\ln\left[1-e^{-{\left(e^{\delta x_{i}^{\beta }}-1\right)}^{2}}\right],\\ \frac{\partial \ell \left(\Omega \right)}{\partial \beta }=\frac{n}{\beta }+\overset{n}{\underset{i=1}{\sum }}\ln\left(x_{i}\right)-2\delta \overset{n}{\underset{i=1}{\sum }}U_{i}+\delta \overset{n}{\underset{i=1}{\sum }}\frac{\ln\left(x_{i}\right)x_{i}^{\beta }e^{-\delta x_{i}^{\beta }}}{1-e^{-\delta x_{i}^{\beta }}}+2\alpha \delta \overset{n}{\underset{i=1}{\sum }}x_{i}^{\beta }\ln\left(x_{i}\right)+4\lambda \alpha \delta \overset{n}{\underset{i=1}{\sum }}\frac{U_{i}e^{-{\left(e^{\delta x_{i}^{\beta }}-1\right)}^{2}}{\left[1-e^{-{\left(e^{\delta x_{i}^{\beta }}-1\right)}^{2}}\right]}^{\alpha -1}{\left\{1-{\left[1-e^{-{\left(e^{\delta x_{i}^{\beta }}-1\right)}^{2}}\right]}^{\alpha }\right\}}^{\lambda -1}}{1+{\left\{1-{\left[1-e^{-{\left(e^{\delta x_{i}^{\beta }}-1\right)}^{2}}\right]}^{\alpha }\right\}}^{\lambda }}-\overset{n}{\underset{i=1}{\sum }}U_{i}e^{-{\left(e^{\delta x_{i}^{\beta }}-1\right)}^{2}}\left\{2\left(\lambda -1\right)\delta \alpha \frac{{\left[1-e^{-{\left(e^{\delta x_{i}^{\beta }}-1\right)}^{2}}\right]}^{\alpha -1}}{1-{\left[1-e^{-{\left(e^{\delta x_{i}^{\beta }}-1\right)}^{2}}\right]}^{\alpha }}+\frac{2\delta \left(\alpha -1\right)}{1-e^{-{\left(e^{\delta x_{i}^{\beta }}-1\right)}^{2}}}\right\},\\ \frac{\partial \ell \left(\Omega \right)}{\partial \delta }=\frac{n}{\delta }-2\overset{n}{\underset{i=1}{\sum }}x_{i}^{\beta }e^{\delta x_{i}^{\beta }}\left(e^{\delta x_{i}^{\beta }}-1\right)+\overset{n}{\underset{i=1}{\sum }}\frac{{x_{i}^{\beta }}^{-\delta x_{i}^{\beta }}}{1-e^{-\delta x_{i}^{\beta }}}+2\overset{n}{\underset{i=1}{\sum }}x_{i}^{\beta }+4\lambda \alpha \overset{n}{\underset{i=1}{\sum }}\frac{W_{i}{\left[1-e^{-{\left(e^{\delta x_{i}^{\beta }}-1\right)}^{2}}\right]}^{\alpha -1}{\left\{1-{\left[1-e^{-{\left(e^{\delta x_{i}^{\beta }}-1\right)}^{2}}\right]}^{\alpha }\right\}}^{\lambda -1}}{1+{\left\{1-{\left[1-e^{-{\left(e^{\delta x_{i}^{\beta }}-1\right)}^{2}}\right]}^{\alpha }\right\}}^{\lambda }}-2\left(\lambda -1\right)\alpha \overset{n}{\underset{i=1}{\sum }}\frac{W_{i}{\left[1-e^{-{\left(e^{\delta x_{i}^{\beta }}-1\right)}^{2}}\right]}^{\alpha -1}}{1-{\left[1-e^{-{\left(e^{\delta x_{i}^{\beta }}-1\right)}^{2}}\right]}^{\alpha }}+2\left(\alpha -1\right)\overset{n}{\underset{i=1}{\sum }}\frac{W_{i}}{1-e^{-{\left(e^{\delta x_{i}^{\beta }}-1\right)}^{2}}}, \end{array}$$

where *U*_*i*_ = ln(*x*_*i*_)*x*_*i*_^*β*^*e*^*δx*_*i*_^*β*^^(*e*^*δx*_*i*_^*β*^^ − 1) and *W*_*i*_ = *x*_*i*_^*β*^*e*^*δx*_*i*_^*β*^^(*e*^*δx*_*i*_^*β*^^ − 1)*e*^−(*e*^*δx*_*i*_^*β*^^ − 1)^2^^.

The numerical solution of such equations, which cannot be obtained from the analysis, may be accomplished by the use of statistical analysis software using iterative approaches.

## 4. Bayesian Estimation

In this section, the Bayesian hypothesis for unknown parameters of both models is constructed by using left censoring in the case of both informative and flat priors in the case of both informative and flat priors. Both of these priors are used. The squared error loss function is something that is taken into consideration (SELF). The next part has an explanation that is more fundamental in nature about the loss function, priors, and the posterior analysis:

In loss function, the loss function $Lo\left(\Omega ,\tilde{\Omega }\right)={\left(\tilde{\Omega }-\Omega \right)}^{2}$ is called SELF, which is the simplest symmetric loss function. The Bayes estimator of *Ω* under SELF is $\tilde{\Omega }=E\left(\Omega \left|X\right.\right)$ with risk *Var*(*Ω*|*X*). In this case, the expectation and variance are calculated in relation to the posterior PDF. Initial applications included estimate issues where an unbiased estimator of *Ω* was being evaluated, and it is still in use today.

The previous distribution that we choose is often determined by the kind of prior information that we have at our disposal. When we have little or no knowledge regarding a parameter, we should utilise a flat prior to estimate it. Previously, a large number of practitioners used flat priors (see Santos and Achcar [26]). When priors are flat, we utilise the gamma distribution to determine baseline parameters $\tilde{\Omega }$. That is, the considered priors PDFs are

(13) $$\begin{array}{c} g\left(\Omega \right)\propto \lambda^{b_{1}-1}e^{-a_{1}\lambda }\alpha^{b_{2}-1}e^{-a_{2}\alpha }\beta^{b_{3}-1}e^{-a_{3}\beta }\delta^{b_{4}-1}e^{-a_{4}\delta },\;\lambda >0,\;\alpha >0,\;\beta >0,\;\delta >0. \end{array}$$

Using the concept of informative priors, the hyperparameters are selected in such a manner that the expectation of each unknown parameter's prior distribution is identical to the actual value. Numerous scientists, notably Chacko and Mohan [27], have employed this strategy to great effect. This section investigates the use of Bayesian estimating to get estimates of the TIHLBW model parameters in order to realize those estimations. As we can see, the maximum likelihood estimate (MLE) approach is very important, yet it is ineffective when dealing with a high-dimensional optimization issue, as we will show. As a result, Bayesian estimation may be more accurate in estimating the parameter than MLEs.

As a result, we merged the likelihood function (10) and joint prior density (13) and used Bayes' theorem to construct the joint posterior density function *Ω* up to a constant.

(14) $$\begin{array}{c} \Pi \left(\Omega \right)\propto \lambda^{n+b_{1}-1}\alpha^{n+b_{2}-1}\beta^{n++b_{3}-1}\delta^{n++b_{4}-1}e^{-a_{1}\lambda -a_{2}\alpha -a_{3}\beta }e^{-\delta \left(a_{4}+-2\overset{n}{\underset{i=1}{\sum }}x_{i}^{\beta }\right)}\times e^{-\overset{n}{\underset{i=1}{\sum }}{\left(e^{\delta x_{i}^{\beta }}-1\right)}^{2}}\overset{n}{\underset{i=1}{\prod }}x_{i}^{\beta -1}\left(1-e^{-\delta x_{i}^{\beta }}\right){\left[1-e^{-{\left(e^{\delta x_{i}^{\beta }}-1\right)}^{2}}\right]}^{\alpha -1}\times \overset{n}{\underset{i=1}{\prod }}{\left\{1-{\left[1-e^{-{\left(e^{\delta x_{i}^{\beta }}-1\right)}^{2}}\right]}^{\alpha }\right\}}^{\lambda -1}{\left\{1+{\left\{1-{\left[1-e^{-{\left(e^{\delta x_{i}^{\beta }}-1\right)}^{2}}\right]}^{\alpha }\right\}}^{\lambda }\right\}}^{-2}. \end{array}$$

It is hard to incorporate out joint posterior distributions because of the high-dimensional integration of joint posterior distributions. As a result, we use the most widely used MCMC approach. The Metropolis-Hastings algorithm, as well as Gibbs samplers, has indeed been implemented in the MCMC approach. In order to determine if a Markov chain is approaching a stable distribution, the Heidelberger-Welch test has been applied. It has been proposed that entire conditional distributions may be generated by multiplying the joint distribution of the model parameter by the joint distribution of the model parameter.

## 5. Simulation Analysis

MCMC is used in this part to execute a Monte Carlo simulation approach to compare the MLEs and the Bayesian estimation method under the condition of self-evaluation (SELF) for estimating the parameters of the TIHLBW distribution. To produce these analyses, we may utilise a variety of software tools such as the Mathcad, Mathematica, Maple, and R packages. Based on data-generated 10000 random samples from TLHLBW distribution, where *x* represents the TIHLBW lifetime, Monte Carlo experiments are carried out for various real values of parameters and varied sample sizes *n* (25, 50, and 100). We might define the best estimator approaches as those that reduce the bias and mean squared error (MSE) of estimators to the greatest extent possible. We make use of several cases of real values, such as in Table 1,

1. actual case I: *λ* = 1.2, *α* = 0.5, *β* = 1.5, and *δ* = 1.5
2. actual case II: *λ* = 1.2, *α* = 2, *β* = 1.5, and *δ* = 1.5
3. actual case III: *λ* = 1.2, *α* = 0.5, *β* = 3, and *δ* = 1.5
4. actual case IV: *λ* = 1.2, *α* = 2, *β* = 3, and *δ* = 1.5

In Table 2,

1. actual case I: *λ* = 3, *α* = 0.5, *β* = 1.5, and *δ* = 0.5
2. actual case II: *λ* = 3, *α* = 2, *β* = 1.5, and *δ* = 0.5
3. actual case III: *λ* = 3, *α* = 0.5, *β* = 3, and *δ* = 0.5
4. actual case IV: *λ* = 3, *α* = 2, *β* = 3, and *δ* = 0.5

The following remarks can be noted from Tables 1 and 2:

1. The bias and MSE decrease in proportion to the increase in sample size
2. When it comes to estimating the parameters of the TIHLBW distribution, the Bayesian technique outperforms the Markov chain method (MLE) in terms of bias and MSE
3. When the value of *α* increases, the bias and MSE for the TIHLBW parameters fall in certain cases

## 6. Applications

In this part, two real-world examples using COVID-19 data from various nations are provided to evaluate the validity of the TIHLBW distribution. The TIHLBW performance in comparison to various similar models, including TIHLB-exp (TIHLBE) [15], TIHLB-Lomax (TIHLBL) [15], odd log-logistic modified Weibull (OLLMW) [28], Kumaraswamy Weibull (KW) [29], generalized modified Weibull (GMW) [30], and Kumaraswamy exponentiated Rayleigh (KER) [31] distributions. Tables 3 and 4 obtained MLE estimates and standard errors (SE) for all parameter of the models. Tables 5 and 6 obtained Kolmogorov-Smirnov distance (KSD) statistic along with its *P* value, CramÃ©r-von Mises value (CVMV), and Anderson-Darling value (ADV) for all models that were calibrated based on two genuine data sets of COVID-19 data with various nations such as Saudi Arabia and Italy, where these data constituted of a drought mortality rate.

### 6.1. Saudi Arabia Data

The first group of information consists of COVID-19 data obtained from Saudi Arabia. These measurements were taken over the course of 37 days, beginning on June 27 and ending on August 2, 2021. The following is the fatality rate that was used to acquire the data: 0.0195, 0.0213, 0.0214, 0.0217, 0.0231, 0.0233, 0.0235, 0.0235, 0.0238, 0.0239, 0.0245, 0.0260, 0.0264, 0.0268, 0.0270, 0.0271, 0.0275, 0.0278, 0.0278, 0.0282, 0.0282, 0.0285, 0.0287, 0.0294, 0.0296, 0.0300, 0.0301, 0.0309, 0.0310, 0.0313, 0.0314, 0.0315, 0.0324, 0.0325, 0.0328, 0.0332, and 0.0358.

### 6.2. Italy Data

The second data set is a COVID-19 data set that belongs to Italy and spans 172 days, from the first of March to the twentieth of August, 2020. The information is as follows: 0.0107, 0.0490, 0.0601, 0.0460, 0.0533, 0.0630, 0.0297, 0.0885, 0.0540, 0.1720, 0.0847, 0.0713, 0.0989, 0.0495, 0.1025, 0.1079, 0.0984, 0.1124, 0.0807, 0.1044, 0.1212, 0.1167, 0.1255, 0.1416, 0.1315, 0.1073, 0.1629, 0.1485, 0.1453, 0.2000, 0.2070, 0.1520, 0.1628, 0.1666, 0.1417, 0.1221, 0.1767, 0.1987, 0.1408, 0.1456, 0.1443, 0.1319, 0.1053, 0.1789, 0.2032, 0.2167, 0.1387, 0.1646, 0.1375, 0.1421, 0.2012, 0.1957, 0.1297, 0.1754, 0.1390, 0.1761, 0.1119, 0.1915, 0.1827, 0.1548, 0.1522, 0.1369, 0.2495, 0.1253, 0.1597, 0.2195, 0.2555, 0.1956, 0.1831, 0.1791, 0.2057, 0.2406, 0.1227, 0.2196, 0.2641, 0.3067, 0.1749, 0.2148, 0.2195, 0.1993, 0.2421, 0.2430, 0.1994, 0.1779, 0.0942, 0.3067, 0.1965, 0.2003, 0.1180, 0.1686, 0.2668, 0.2113, 0.3371, 0.1730, 0.2212, 0.4972, 0.1641, 0.2667, 0.2690, 0.2321, 0.2792, 0.3515, 0.1398, 0.3436, 0.2254, 0.1302, 0.0864, 0.1619, 0.1311, 0.1994, 0.3176, 0.1856, 0.1071, 0.1041, 0.1593, 0.0537, 0.1149, 0.1176, 0.0457, 0.1264, 0.0476, 0.1620, 0.1154, 0.1493, 0.0673, 0.0894, 0.0365, 0.0385, 0.2190, 0.0777, 0.0561, 0.0435, 0.0372, 0.0385, 0.0769, 0.1491, 0.0802, 0.0870, 0.0476, 0.0562, 0.0138, 0.0684, 0.1172, 0.0321, 0.0327, 0.0198, 0.0182, 0.0197, 0.0298, 0.0545, 0.0208, 0.0079, 0.0237, 0.0169, 0.0336, 0.0755, 0.0263, 0.0260, 0.0150, 0.0054, 0.0375, 0.0043, 0.0154, 0.0146, 0.0210, 0.0115, 0.0052, 0.2512, 0.0084, 0.0125, 0.0125, 0.0109, and 0.0071.

It is evident from Tables 3 and 4 that the TIHLBW, TIHLBE, TIHLBL, KS, OLLMW, and GMW distributions have MLE and SE estimations. In addition, the *P* value for KS is maximum for the TIHLBW distribution (see Tables 5 and 6). In addition, the KSD, CVMV, and ADV have their lowest values for the TIHLBW distribution as compared to other models (see Tables 5 and 6). Since demonstrated in Figures 3 and 4, the four roots of the parameters in the COVID-19 data sets are all global maximums, which indicates that the data sets perform rather well. We drew the log by establishing two parameters and adjusted the others. Figures 5 and 6 show the probabilities for each parameter in COVID-19 data sets. This leads us to the conclusion that the TIHLBW distribution is a superior match for the three actual data sets from Saudi Arabia and Italy. The estimated PDF of model plots provided in Figures 7 and 8 demonstrates that our distribution is a good fit for modelling the COVID-19 data presented above.

## 7. Major Findings and Conclusions

During the course of this research, the idea of developing and researching a new Weibull distribution that is based on the type I half logistic Burr *G* family was brought up, and it was studied. In order to make an accurate estimates of the unknowable parameters included in this investigation, the methodologies of maximum likelihood and Bayesian estimation were used. The TIHLBW distribution provides a better match than other submodels, including the TIHLB-exp distribution, the TIHLB-Lomax distribution, the odd log-logistic modified Weibull distribution, the Kumaraswamy Weibull distribution, the generalized modified Weibull distribution, and the Kumaraswamy exponentiated Rayleigh distributions. An R software was used in order to carry out a simulation research so that a comparison could be made about how well the different methods of estimation worked. The MCMC methodology was used in order to arrive at a Bayesian estimate of the data. Two sets of real-world COVID-19 data from a variety of countries, such as Italy and Saudi Arabia, were taken into account. For more reading, see [19, 32–42].

## 8. Future Work

The expansion of classical statistics is known as neutrophilic statistics, and it is applicable to situations in which the data in question originates from a complex issue or an unpredictable context. Our present work may be expanded using neutrosophic statistics as future research, and we will use the preceding publications as sources and guides in our future studies. In addition, our present project can be improved utilising neutrosophic statistics.

The future effort will include us applying the suggested distribution as well as the newly established family of distributions to the censored sample method. We are going to experiment with several types of censoring schemes, and we are going to produce random censored samples based on the new distribution. Our research may be expanded to include the application of the suggested model to several kinds of accelerated life testing, and perhaps even progressive load accelerated life test results. In the end, we are going to apply a variety of different optimality criteria to the censored samples that were created by the suggested model. For more reading, see Ramzan et al. [43].

## Figures and Tables

**Figure 1:** PDF TIHLBW model.

**Figure 2:** HR function of TIHLBW model.

**Figure 3:** Profile-likelihood for the four parameters for COVID-19 data of Saudi Arabia.

**Figure 4:** Profile-likelihood for the four parameters for COVID-19 data of Italy.

**Figure 5:** Contour plot for log-likelihood for COVID-19 data of Saudi Arabia.

**Figure 6:** Contour plot for log-likelihood for COVID-19 data of Italy.

**Figure 7:** Fitted CDF with empirical CDF, estimated PDF, and P-P plots for COVID-19 data of Saudi Arabia.

**Figure 8:** Fitted CDF with empirical CDF, estimated PDF, and P-P plots for COVID-19 data of Italy.

**Table 1:** MLE and Bayesian estimation for parameter of TIHLBW distribution when *λ* = 1.2,  *δ* = 1.5 and other values.

*λ* = 1.2, *δ* = 1.5			*α* = 0.5				*α* = 2			
			MLE		Bayesian		MLE		Bayesian	
*β*	*n*		Bias	MSE	Bias	MSE	Bias	MSE	Bias	MSE
1.5	25	*λ*	0.0264	0.2286	0.0464	0.0137	-0.1535	0.0847	0.0516	0.0163
		*α*	0.1282	0.3086	0.0547	0.0409	-0.0272	0.9604	0.0448	0.1072
		*β*	0.3121	0.8010	0.1202	0.0734	0.4296	0.9017	0.1031	0.0413
		*δ*	0.3520	0.5737	0.0374	0.0129	0.3031	0.3551	0.0412	0.0103
	50	*λ*	0.0533	0.2235	0.0451	0.0126	-0.1547	0.0802	0.0478	0.0154
		*α*	0.0597	0.1364	0.0445	0.0283	0.0787	0.7540	0.0296	0.1017
		*β*	0.2275	0.5454	0.1039	0.0653	0.2111	0.3269	0.0909	0.0351
		*δ*	0.1855	0.2008	0.0327	0.0112	0.1785	0.0939	0.0373	0.0084
	100	*λ*	0.0281	0.1606	0.0355	0.0118	-0.0561	0.0224	0.0430	0.0123
		*α*	0.0201	0.0531	0.0256	0.0208	-0.0250	0.3409	0.0351	0.1005
		*β*	0.1229	0.2551	0.0911	0.0574	0.1235	0.1309	0.0770	0.0315
		*δ*	0.1020	0.0912	0.0306	0.0102	0.0684	0.0201	0.0303	0.0060
3	25	*λ*	0.1136	0.3861	0.0386	0.0147	-0.1945	0.1197	0.0463	0.0152
		*α*	0.1382	0.2610	0.0586	0.0288	0.0663	0.7905	0.1304	0.1354
		*β*	0.1726	1.2476	0.0542	0.0324	0.4725	1.0935	0.0925	0.0425
		*δ*	0.2043	0.3312	0.0275	0.0118	0.2321	0.1737	0.0272	0.0072
	50	*λ*	0.0933	0.3041	0.0342	0.0124	-0.0889	0.0642	0.0299	0.0148
		*α*	0.0442	0.0808	0.0415	0.0173	0.1793	0.5747	0.0854	0.1022
		*β*	0.1985	0.8358	0.0527	0.0313	0.1391	0.3592	0.0834	0.0406
		*δ*	0.1253	0.1636	0.0227	0.0080	0.0871	0.0306	0.0280	0.0063
	100	*λ*	0.0317	0.2076	0.0341	0.0119	-0.0769	0.0351	0.0195	0.0132
		*α*	0.0174	0.0318	0.0296	0.0112	0.0736	0.3362	0.0550	0.1000
		*β*	0.0649	0.3402	0.0507	0.0305	0.1150	0.2968	0.0733	0.0406
		*δ*	0.0749	0.0787	0.0166	0.0068	0.0625	0.0198	0.0284	0.0050

**Table 2:** MLE and Bayesian estimation for parameter of TIHLBW distribution when *λ* = 3, *δ* = 0.5 and other values.

*λ* = 3, *δ* = 0.5			*α* = 0.5				*α* = 2			
			MLE		Bayesian		MLE		Bayesian	
*β*	n		Bias	MSE	Bias	MSE	Bias	MSE	Bias	MSE
1.5	25	*λ*	-0.2111	0.4032	0.0063	0.0030	-0.0026	0.0006	0.0014	0.0003
		*α*	0.0876	0.1568	0.0535	0.0274	0.0317	0.0907	0.0259	0.0851
		*β*	0.2663	0.5802	0.1483	0.0908	0.1040	0.0912	0.1012	0.0564
		*δ*	0.0550	0.0233	0.0078	0.0061	-0.0081	0.0026	-0.0078	0.0019
	50	*λ*	-0.0977	0.1410	0.0061	0.0030	-0.0020	0.0002	0.0012	0.0002
		*α*	0.0497	0.0674	0.0468	0.0235	0.0101	0.0441	0.0093	0.0390
		*β*	0.1061	0.2411	0.1044	0.0898	0.0387	0.0339	0.0288	0.0315
		*δ*	0.0245	0.0095	0.0043	0.0046	-0.0040	0.0012	-0.0013	0.0011
	100	*λ*	-0.0668	0.0901	0.0059	0.0029	-0.0004	0.0002	0.0002	0.0002
		*α*	0.0372	0.0480	0.0344	0.0193	0.0005	0.0282	0.0003	0.0182
		*β*	0.0871	0.1970	0.0870	0.0880	0.0280	0.0223	0.0190	0.0148
		*δ*	0.0122	0.0058	-0.0022	0.0039	-0.0032	0.0008	-0.0021	0.0007
3	25	*λ*	-0.2365	0.5905	0.0128	0.0027	-0.0011	0.0016	0.0146	0.0013
		*α*	0.0395	0.0794	0.0347	0.0175	0.0743	0.1037	0.1039	0.0939
		*β*	0.1953	0.5684	0.0607	0.0321	0.0836	0.1205	0.0789	0.0409
		*δ*	0.0632	0.0214	0.0079	0.0046	0.0003	0.0014	-0.0039	0.0009
	50	*λ*	-0.0707	0.1302	0.0140	0.0023	0.0008	0.0004	0.0004	0.0003
		*α*	0.0150	0.0139	0.0131	0.0082	0.0260	0.0457	0.0175	0.0392
		*β*	0.0733	0.1324	0.0656	0.0304	0.0412	0.0517	0.0407	0.0406
		*δ*	0.0231	0.0048	0.0078	0.0028	-0.0007	0.0006	-0.0006	0.0005
	100	*λ*	-0.0624	0.1274	0.0082	0.0021	-0.0005	0.0003	0.0001	0.0003
		*α*	0.0120	0.0117	0.0120	0.0050	0.0122	0.0290	0.0105	0.0183
		*β*	0.0246	0.1187	0.0225	0.0248	0.0154	0.0327	0.0566	0.0254
		*δ*	0.0196	0.0031	0.0050	0.0017	0.0003	0.0004	-0.0027	0.0003

**Table 3:** MLE for Saudi Arabia data.

		*λ*	*α*	*β*	*δ*
TIHLBW	Estimates	48.1999	2.1852	1.4615	67.4952
	SE	0.0069	0.0043	0.0022	0.0045
TUHLBE	Estimates	14.1517	3.6447	0.0467	
	SE	33.0825	0.8766	0.0188	
TIHLBL	Estimates	1.3570	6.4543	0.5680	19.7100
	SE	2.4011	5.5973	1.9628	66.2191
KS	Estimates	3.9925	12.4107	31.0745	2.8601
	SE	24.8132	127.4390	21.8936	13.7647
OLLMW	Estimates	10.5314	6.7451	7.5742	0.7531
	SE	12.2575	73.7284	10.2987	0.5212
GMW	Estimates	79.1348	7.7471	62.7334	1.4464
	SE	20.1560	9.0892	34.6153	0.3317

**Table 4:** MLE for Italy data.

		*λ*	*α*	*β*	*δ*
TIHLBW	Estimates	1.1716	0.8199	0.5148	1.8929
	SE	1.2784	0.2916	0.1814	0.4230
TUHLBE	Estimates	6.0662	0.5177	0.7225	
	SE	4.3622	0.0653	0.2938	
TIHLBL	Estimates	1.4204	0.4813	0.2133	1.0133
	SE	0.9456	0.1517	0.1549	0.8522
OLLMW	Estimates	20.7185	0.3096	0.6924	0.0249
	SE	12.7877	0.2029	0.0147	0.0162
KS	Estimates	0.4471	0.3428	9.5106	2.0612
	SE	0.1097	0.0813	0.9027	0.2006
GMW	Estimates	2.6124	5.9942	3.0918	0.2462
	SE	0.7070	8.4543	0.8185	0.2231
KER	Estimates	105.2955	0.5725	24.8535	0.0207
	SE	69.6219	0.3307	13.0358	0.0109

**Table 5:** Goodness-of-fit measures for Saudi Arabia data.

	KSD	P-V.KS	CVMV	ADV
TIHLBW	0.0936	0.8723	0.0362	0.2607
TUHLBE	0.0980	0.8351	0.0379	0.2827
TIHLBL	0.0998	0.8190	0.0412	0.2847
KS	0.1006	0.8118	0.0379	0.2692
OLLMW	0.1124	0.6964	0.0791	0.5046
GMW	0.0942	0.8671	0.0541	0.3458

**Table 6:** Goodness-of-fit measures for Italy data.

	KSD	P-V.KS	CVMV	ADV
TIHLBW	0.0501	0.7773	0.1179	0.7285
TUHLBE	0.0587	0.5901	0.1436	0.8437
TIHLBL	0.0529	0.7175	0.1209	0.7339
OLLMW	0.0604	0.5526	0.2184	1.3017
KS	0.0527	0.7230	0.1195	0.7308
GMW	0.0621	0.5163	0.1511	0.8802
KER	0.0712	0.3443	0.1715	0.9792

## Data Availability

The data is attached to this paper.
